This article has been retracted.

# Effect of Micropower Vacuum Dressing on Promoting Wound Healing in Patients with I-II Diabetic Foot

**DOI:** 10.1155/2022/2577601

**Published:** 2022-05-06

**Authors:** Cunren Chen, Xixiong Wang, Changli Liang, Haiwei Liu

**Affiliations:** ^1^Department of Endocrinology, Hainan General Hospital, Hainan Affiliated Hospital of Hainan Medical University, Haikou 570311, Hainan, China; ^2^Department of Breast Surgery, Boao Yiling Life Care Center, Qionghai 571400, Hainan, China

## Abstract

**Objective:**

Discuss the effectiveness and value of micropower vacuum dressing (MVD) in promoting the healing of I-II grades diabetic foot wounds.

**Methods:**

Sixty patients diagnosed with diabetic foot ulcers and Wagner grades I-II were selected and randomly divided into the control group and experimental group, with 30 cases in each group. The control group was covered with conventional treatments and petrolatum gauze dressings, and the experimental group was treated with MVD on the basis of conventional reatments. The therapeutic effects of the two groups were observed, including healing rate, ulcer area reduction rate, ulcer healing time, dressing change times, ulcer recurrence rate, adverse events, and so on.

**Results:**

The healing rate (100%) of the experimental group was higher than that of the control group (56.7%); the wound reduction rate was higher than that of the control group (*P* < 0.05); the healing time, the number of dressing changes, and the 1-month recurrence rate were all low in the control group (*P* < 0.05). The incidence of adverse reactions in the experimental group (6.7%) was lower than that in the control group (46.7%) (*P* < 0.05).

**Conclusion:**

MVD has significant effects in the treatment of I-II grades diabetic foot wounds and has few adverse reactions. It is an effective new method that can promote the growth of granulation tissue and epithelium and promote wound healing.

## 1. Introduction

Diabetes mellitus (DM) is a group of metabolic diseases characterized by hyperglycemia [1]. Diabetes is a serious health problem. The long-term complications of hyperglycemia include heart disease, stroke, diabetic retinopathy, and peripheral neuropathy. Diabetic foot infection, ulceration, and deep tissue destruction due to nerve abnormalities and varying degrees of vascular lesions in the distal part of the lower extremities may result in surgical debridement or amputation. It is estimated that up to 20% of diabetic foot patients need hospitalization. Epidemiological studies show that the risk of foot ulcers is 2.5% per year [2].

Treatment of diabetic foot infections requires careful wound management, good nutrition, proper use of antimicrobial agents, good glycemic control, and maintenance of fluid and electrolyte balance. Although patients with severe infections need to be hospitalized for surgical emergency consultation, antibacterial treatment, and stabilize the condition, most mild infections and many moderate infections can be treated in the outpatient department and closely followed up. A number of studies have reported the use of multidisciplinary combined treatment to improve the incidence of diabetic foot infection, including wound care, infectious diseases, endocrinology, and surgical professionals [3]. The principle of micropower vacuum dressing is similar to that of closed negative pressure, but it can be used as a supplement to closed negative pressure because of its small pressure.

Micropower vacuum dressing (MVD) is the use of special materials to produce the “siphon effect” and “pump effect,” form micronegative pressure, and promote wound healing [4]. At present, this method has been widely applied to burn wounds in burn department, but it has not been applied in the treatment of diabetic foot wounds. My department is effective in treating Wagner grades I-II foot diabetic foot wounds with this dressing and is more convenient in operation for other traditional dressings. It not only shortens the hospital stay but also reduces the amount of labor for medical staff. This study further confirmed the effect of micropower vacuum dressing in the treatment of diabetic foot by comparing clinical observation with a view to exploring an alternative method for the treatment of diabetic foot.

## 2. Methods

### 2.1. Participants

A convenience sample of 60 participants enrolled in this investigation. Participants were directly recruited from a bone health clinic in a Hainan Provincial People's Hospital. The severity of diabetic foot was classified according to Wagner grading standard. Grade 0: there are risk factors for ulcer, but there is no ulcer; grade I: superficial ulcer, no infection; grade II: deep ulcer and fascia, but no abscess and bone involvement; grade III: deep ulcer with abscess formation, bone involvement to osteomyelitis; grade IV: localized gangrene; grade V: gangrene in all feet.

The inclusion criteria for participation were in line with the diagnostic criteria for diabetes and diabetic foot (Wagner classification, I-II grades) in type 2 diabetes patients aged 20–80 years (male or female) and HbA1C 7.0–16% in 2016 WHO. The exclusion criteria were diabetic foot (Wagner grade, III–V grades), specific infection wounds (tuberculosis and tetanus wounds), diabetes mellitus complicated with ketoacidosis and hypertonic coma, severe heart, liver, and kidney dysfunctions, those treated with glucocorticoids, and ankle brachial index (ABI) <0.7. All participants were recruited and screened for eligibility by a physician from our hospital who has professional qualification certificate. The study was approved by the hospital's institutional review board. The patients were randomly divided into the control group and experimental group, with 30 cases in each group. The control patients had similar characteristics (i.e., sex, ethnicity, age, chief complaint, comorbidities, and admission time) to the patients in the experimental group.

### 2.2. Research Design

The control group received routine treatment including smoking cessation liquor, diabetes diet, improving microcirculation, nutritional nerve, anti-inflammatory, and systemic nutritional status, monitoring blood glucose level and local wound debridement and dressing, and vaseline gauze dressing. The dressing change times are determined according to the amount of liquid seepage. The dressing can be changed once in 1-2 days in the initial stage and 2-3 days in the later stage. The experimental group was covered with MVD (composed of special polyvinyl alcohol medical materials with high water absorption and medical transparent adhesive film, which is purchased from Guangzhou Meijie Weitong Biotechnology Co., Ltd.) on the basis of routine treatment. The finger pressure method is used to judge the saturation of the dressing. If the dressing is saturated, it can be replaced in time. It can be placed for 2-3 days at the shortest time and 5–7 days at the longest time.

### 2.3. Detection Index

① Complete healing rate of target ulcer: it refers to the percentage of cases with complete healing of target ulcer in the total number of cases in the human group within 4 weeks of treatment. The criterion of complete healing of ulcer is skin epidermal cell regeneration and no secretion or dressing requirements. ② Ulcer area reduction rate: the ulcer area was evaluated in the second week. Measurement of wound area: cover the wound with a piece of sterile transparent film, including the concave part, draw a circle along the edge with a marker pen, take out the transparent film, flatten the transparent film, and measure the scribed area. Digital photography and macrofocusing were used to take vertical photos of the ulcer surface and import it into the computer. The wound area = length calculated by Image J image analysis software × wide. Reduction rate of ulcer area = (baseline ulcer area − ulcer area in this follow-up)/baseline ulcer area × 100%. ③ Complete healing time: it refers to the time required for healing if the target ulcer surface is completely covered by new epithelial tissue. ④ Dressing change times. ⑤ Recurrence rate: patients with complete ulcer healing continue to be followed up for 1 month. Pay attention to the number of cases with recurrence and distinguish between real wound closure and temporary wound coverage.

Comparison of adverse reactions: the number of cases of bleeding, pain, and swelling.

### 2.4. Data Analysis

The obtained data were statistically analyzed by SPSS statistics (version 22), and the continuous variables were analyzed by the *t*-test. Counting data use the *λ*2 test, *P* < 0.05 means the difference is statistically significant.

## 3. Results

### 3.1. Basic Demographic and Clinical Characteristics

There were no differences between the two groups, including for wound surface area, history of major and minor amputations, and ankle brachial index (ABI). The erroneously normal values for ABI probably reflected the stiff calcified vessels in the diabetic and renal patients (Table 1).

### 3.2. Comparison of Clinical Efficacy between the Two Groups

The healing rate of the experimental group (100%) was higher than that of the control group (56.7%). After 2 weeks of initial treatment, the wound shrinkage rate was higher than that in the control group (*P* < 0.05). The healing time, dressing change times, and 1-month recurrence rate in the control group were lower than those in the control group (*P* < 0.05) (Table 2, Figure 1).

### 3.3. Comparison of Adverse Reactions between the Two Groups

In the experimental group, there were 0 cases of bleeding, 0 cases of pain, 2 cases of redness and swelling, and the incidence of adverse reactions was 6.7%. In the control group, there were 6 cases of bleeding, 7 cases of pain, and 6 cases of redness and swelling. The incidence of adverse reactions was 46.7%. The incidence of adverse reactions in the experimental group was significantly higher than that in the control group (*P* < 0.05) (Table 3).

## 4. Discussion

Diabetic foot disease is one of the most serious chronic complications of diabetes. It is not only difficult to treat but also expensive and time-consuming. The annual incidence of ulceration for DM patients and amputation for diabetic foot ulcer patients were 8.1 and 5.1%, respectively [5, 6].

In this study, the healing rate of the experimental group (100%) was higher than that of the control group (56.7%). After 2 weeks of initial treatment, the wound shrinkage rate was higher than that in the control group (*P* < 0.05). The healing time, dressing change times, and 1-month recurrence rate in the control group were lower than those in the control group. It indicates that MVD can effectively improve wound reduction, shorten healing time, reduce dressing change times, and promote wound healing in patients with I-II class diabetic foot. At the same time, after one month of wound healing, the experimental group achieved zero relapse, and the recurrence rate was significantly reduced compared with the control group. At present, the treatment of wound advocates the “wet healing” theory, which refers to creating a slightly acidic and slightly wet environment for the local part of the wound, which is more in line with the physiological state, so as to promote wound angiogenesis, granuloma formation, and epidermal proliferation and finally achieve effective wound healing. Vacuum sealing drainage (VSD) keeps continuous drainage of wound exudates, avoids bacterial residue in the wound, controls infection, and reduces granulation edema. It explains the reliability of the theory of “moist healing” in all directions and has been widely used in the treatment of diabetic foot, and its curative effect has been recognized [7, 8].

Diabetic foot Wagner I level refers to superficial ulcers of the feet, no signs of infection, and prominent manifestations of nerve ulcers. Grade II refers to deep ulcer, often complicated with soft tissue infection and without osteomyelitis or deep abscess. These two kinds of wounds mainly control infection, control exudation, and promote granulation growth and skin crawling. Due to the high negative pressure, the atmospheric pressure produced by closed negative pressure drainage can compress and stimulate local wounds, which is not conducive to the growth and crawling of epithelium [9]. The application of these two kinds of wounds has been limited to a certain extent. However, the principle of MVD is similar to closed negative pressure, but it can be used as a better supplement to closed negative pressure because of its small pressure. In addition, the wound treatment of Wagner grades I-II is mainly based on foam dressing. Although the dressings have some functions of absorbing and moisturizing, because of its limited function of absorbing water, if they are not replaced in time, the wound exudate cannot be effectively controlled. Not only can bacteria be easily propagated and infected but also the biofilm is easily formed, thus impeding cell growth [10, 11]. The traditional dressing did not promote the growth of granulation and epithelium. Although some skin defect wounds can be healed by skin grafting, they often cause ulcer recurrence due to poor wear resistance. Only functional repair can be completed by crawling, self sealing, and finally keratinization of the skin around the wound itself. MVD is a new type of dressing for wound treatment. Because its material has strong liquid absorption performance, it can quickly inhale into the material when liquid or blood seeps into contact with the material, forming a “siphon effect” [12]. In addition, because the outer layer is covered with a unidirectional transparent film, when the liquid flows into the surface tension formed by the material, a micronegative pressure is formed locally, resulting in the “pump effect.” A certain humidity can be maintained in this sealed microenvironment, which is conducive to the crawling of epithelial cells and the closure of wounds [13]. Compared with traditional dressings, it has more advantages in absorbing exudates, reducing bacterial residues, controlling infection, destroying the formation of biofilm, reducing edema, creating a wet environment, improving microcirculation, and promoting epithelial growth [14]. At present, the dressing has been widely used in burn wound treatment in burn department [3], but it has not been applied in the treatment of diabetic foot wounds. During the treatment, there were 0 cases of bleeding, 0 cases of pain, and 2 cases of redness and swelling in the experimental group. The incidence of adverse reactions was 6.7% and 46.7%. The difference was statistically significant. It indicates that vacuum sealing drainage combined with microdynamic negative pressure dressing can effectively reduce the incidence of adverse reactions in patients with grades I-II diabetic foot. There was no bleeding and pain during the treatment of the dressing, but there were 2 cases of redness and swelling. Considering that the dressing was not replaced in time, the dressing was over saturated and the wound was soaked, resulting in redness and swelling. After closely monitoring the dressing, there was no redness and swelling after replacing the dressing in time.

In summary, MVD is different from other traditional dressings. It uses the action principle of micronegative pressure to achieve wound healing. It is an innovation in wound treatment at present. Our department is effective in the treatment of diabetic foot wounds with Wagner grades I-II diabetic foot. It can effectively improve the wound reduction rate, shorten the healing time, reduce the frequency of dressing change, promote wound healing, and reduce the recurrence rate after one month. Moreover, in terms of operation, it should be more convenient for other traditional dressings and suitable for out of hospital sequential treatment, which not only shortens the hospital stay but also greatly reduces the labor burden of medical staff.

The deficiency of this study is that the sample size is small and the research is not thorough enough. In the follow-up study, we expanded the sample size and studied the related mechanisms of promoting healing in order to explore a more effective method for the treatment of diabetic foot.

## Figures and Tables

**Figure 1:** Clinical outcome. (a) Just hospitalized. (b) After debridement. (c) After treatment with MVD. (d) 3 days after treatment. (e) 15 days after treatment. (f) 30 days after treatment. (g) Followed up for 1 month.

**Table 1:** Comparison of general information between the two groups.

	Experience group	Control group	*t*/*χ*^2^	*P*
Gender (male/female, no.)	16/14	15/15	0.067	0.796
Age, mean (SD), years	51.47 ± 13.13	52.33 ± 12.54	−0.262	0.795
Ulcer duration ($\bar{x}\pm s$, *d*)	12.17 ± 6.37	13.63 ± 6.22	−0.902	0.371
Ulcer surface area (cm^2^)	16.12 ± 5.23	17.17 ± 5.66	−0.748	0.458
C-reactive protein (mg/L)	7.40 ± 4.10	8.17 ± 4.40	−0.699	0.488
HbA1C ($\bar{x}\pm s$, %)	9.69 ± 1.93	10.17 ± 2.04	−0.936	0.353
Insulin injection	13 (52.0)	12 (48.0)	0.069	0.793
Combined with neuropathy	15 (46.9)	17 (53.1)	0.067	0.796
ABI, mean (SD)	1.01 ± 0.15	0.97 ± 0.12	1.130	0.263
Wagner classification				
I	14 (51.9)	13 (48.1)	0.067	0.795
II	16 (48.5)	17 (51.5)		

**Table 2:** Comparison of treatment conditions between the two groups.

Group	*n*	Healing rate (%)	Reduction rate (%)	Healing time (*d*)	Dressing change times	1-month recurrence rate (%)
Experience group	30	100	82.90 ± 21.18	15.27 ± 6.84	4.73 ± 1.89	0.0
Control group	30	56.7	60.60 ± 25.76	28.20 ± 12.76	13.57 ± 5.59	30.0
*t*/*χ*^2^		14.14^*∗*^	3.662^*∗∗*^	−4.893^*∗∗*^	−8.193^*∗∗*^	8.366^*∗*^
*P*		0.001	0.001	<0.001	<0.001	0.004

**Table 3:** Comparison of adverse reactions.

Group	*n*	Hemorrhage (*n*)	Pain (*n*)	Redness and swelling (*n*)	Incidence of adverse reactions (%)
Experience group	30	0	0	2	6.7
Control group	30	6	7	6	46.7
*χ* ^2^		4.630	5.822	1.298	10.313
*P*		0.031	0.016	0.255	0.001

## Data Availability

The data used to support the findings of this study are available from the corresponding author upon request.
